# Blockchain Powered Vaccine Efficacy for Pharma Sector

**DOI:** 10.1155/2022/4862742

**Published:** 2022-09-10

**Authors:** Sharmila, Shashi Bhushan, Pramod Kumar, Anuj Kumar Garg, Shyam Nair

**Affiliations:** ^1^Department of Electronics & Communication Engineering, Krishna Engineering College, Ghaziabad, India; ^2^Department of Computer Science, Amity University Punjab, Mohali, India; ^3^Department of Computer Science & Engineering, MIET College, Meerut, India; ^4^Department of Blockchain, Zebpay, India; ^5^Department of Information Technology, BlueCrest University College, Liberia

## Abstract

Infectious and contagious diseases exist in humanity for many centuries which causes a curb in the growth of the population. Immunization plays a vital role to prevent mortality and morbidity against infectious diseases. COVID-19 pandemic continues to rage the urgency of developing a vaccine that should ensure the safety, efficacy, swift and fair deployment, implementation, and monitoring of vaccines across the globe. In the present context, the vaccine production to immunization campaign is a critical challenge. Therefore, an effective vaccine supply chain mechanism is required to address issues such as counterfeit vaccines, reduce vaccine wastages, and vaccine record fraud. In this paper, a blockchain-enabled vaccine supply chain is proposed to ensure the correctness, transparency, trust, and immutable log and improve the efficiency of vaccine distribution in the cold chain. The uniqueness of the proposed system is to provide distributed system to verify the reliability and efficacy of the vaccine from production to end beneficiaries' feedback about the vaccine. Our proposed system gives a clear view to the users as well as to the healthcare provider about the vaccination and ensures the anticounterfeit vaccine. The proposed system minimizes counterfeit vaccines and records, provides transparent communication between stakeholders in the supply chain, and improves the security of the vaccine supply chain and immutable feedback system about the vaccine.

## 1. Introduction

Vaccine plays a vital role in the medical field for preventing mortality and morbidity against various infectious diseases. Immunization is related to the safety of public health and the welfare of the nation. Vaccine production as a part of the pharmaceutical industry is involved in the activities of research and development, manufacturing, sales or marketing, and distribution of vaccines. Even during this modern digitalized era, vaccination facilities are outreach in undeveloped countries such as Nigeria [1, 2]. Immunization is a challenging prospect in healthcare, according to a vaccine report [3]. A total share of 37.1% of global storage unit was in low-income countries and 33.3% in high-income countries that were not preserved the vaccine under recommended temperature ranges.

Since the 1980s, a wide range of vaccines are available against diseases such as measles, polio, hepatitis B, pneumonia, rotavirus, and pertussis which have resulted in a reduction in childhood mortality worldwide. Effective vaccine management plays a crucial role due to the cost involved in the production of the vaccines. Traceability and the fight against counterfeit vaccines is an important concern that needs to be managed because of the availability of pseudo/fake vaccines. The National Medical Products Administration (NMPA) is responsible for approving a qualified vaccine that has been verified by various randomized controlled trials (RCTs) [4–7]. In the real world, the supplier makes a profit in an attempt to elude the assessment to measure the effectiveness and safety of the vaccine thereby curbing the cost of research and development and manufacturing which leads to great harm to society. In 2018, the second largest rabies manufacturing company Changchun Changsheng in China violated the regulations while manufacturing 250,000 doses of rabies vaccines which cause serious adverse effects like even blindness reported by more than 50,000 vaccinators. According to the inquiry report submitted by SDA, Changchun Changsheng violated the good manufacturing practices (GMP) by freeze-dried rabies vaccine, fake packaging, and also falsified vaccine records [5].

One of the most serious frauds in medical history was Wakefield fraud [8–11]. Opet et al. discussed the Andrew Wakefield fraud allegation on the measles, mumps, and rubella (MMR) vaccine which caused the risk of autism after vaccination. After the false allegation, MMR vaccination rates began to drop because parents were much more worried about the risk of autism after vaccination. In 2008 and 2009, measles outbreaks in the UK, as well as the USA, were related to the nonvaccination of children [11–17].

In 2003, the Government Primary Health Center in Thiruvananthapuram, India, administrated insulin instead of the hepatitis B vaccine for children. After vaccination, children who complained of giddiness were rushed to the government hospital. In the Inquiry report, it was stated that the hospital administration had procured large quantities of hepatitis B vaccine from three private pharma companies when there was no requirement and also no storage facility to store vaccine vials. Hepatitis B vaccines were stored along with insulin and administrated to children mistakenly [7].

The outbreak of the pandemic SARS-CoV-2 (COVID-19) [8–10] resulted in high mortality and morbidity globally. It urged the development of effective vaccines which should be affordable, safe, swift, and rational deployment. During the COVID-19 pandemic, many immunization companies such as Covishield, Covaxin, Pfizer, and Moderna developed and deployed their vaccine in the market to save the public from COVID-19 infection.

In November 2020, the vaccine was approved for use in a different part of the world; however, there are numerous hurdles with the impact of the implementation of the COVID-19 immunization program [20–25]. Another vaccine fraud was reported recently in India when the number of COVID-19 positive cases across the State increased, and parents were rushed to the hospital to get their school-aged child vaccinated by providing false age. The current monitoring system has failed to detect the counterfeit vaccine package tracking and traceability. Therefore, a novel system is required to improve transparency, traceability, and creditability. The health and pharmaceutical industries have already adopted digitization.

In the current COVID-19 immunization, the vaccine-administrated details are stored in one location which is highly vulnerable to manipulation, tampering, and hacking. Apart from the above issue, there is no review system available for the determination of vaccine efficacy and postvaccination impact on human health.

Recently, NCBI study reported that over $75 billion in revenue is generated annually from anticounterfeit drugs which drastically affects the revenue of the pharmaceutical industry [26]. The aforementioned issues can be addressed with the help of using an effective supply chain management system for monitoring and implementing of vaccination program.

The main contribution of this paper is to address the above issues related to vaccines through blockchain and the Internet of Things. The theme of the paper is as follows:

- The decentralized smart contract-based vaccine monitoring system to ensure the proper vaccine transportation conditions in a cold chain supply, transparent and tamper-proof vaccine administration, reporting of postvaccination side effects, tamper-proof rating, and feedback of vaccination provided by vaccinator
- The rating system is defined based on postvaccination reactions in users such as fever, allergic reaction, irritability, malaise, and swelling
- Recent studies have pointed out the possibilities of using blockchain in COVID-19 vaccine distribution but have not addressed the other types of vaccine (inactivated vaccine, live attenuated vaccine, RNA vaccine, etc.), core vaccine, and noncore vaccine for animals. This paper offers the solutions for reducing vaccine wastage, anticounterfeit, traceability, the authenticity of vaccines, public reporting system, efficiency, transparency, availability, etc.

The rest of this paper is structured as follows: Section 2 discusses the issues and existing work related to the vaccine supply chain. Section 3 presents the proposed blockchain-based vaccine supply chain system. Section 4 summarizes the security analysis of the proposed system. In the end, Section 5 provides the conclusion and future scope of the paper.

## 2. Literature Review

This section summarizes the anticounterfeiting and traceability models available for the vaccine supply chain using new technologies. Information and communication technologies (ICT) offer the way for herd inoculation campaigns for well distribution and planning of vaccines [2–4]. Wallace et al. [1] discussed planning and feasibility assessment facilities through a vaccination simulation tool [31]. In [32, 33], equity constraint-based mathematical modeling was discussed to address vaccine distribution for the heterogeneous population. In [34–36], several heuristics and custom optimization methods are proposed for distributed network design.

Recent advancements in modern technologies such as machine learning, the Internet of Things (IoT) [57–59], and blockchain facilitate a new way of building smart and novel systems for different domains. Kalla et al. [24] discussed the use of IoT technology to monitor the temperature, humidity, and location of logistics to ensure transparency as well as increase immunization coverage in remote areas.

Blockchain technology is integrated with IoT to overcome the gaps between the actual needs and technical limitations. The blockchain eradicates the data storage challenges and ethical issues (confidentiality and privacy of patient health information) addressed by a centralized management mechanism.

In the pharma supply chain, the Internet of Things (IoT) plays a vital role to distribute the vaccine safely and effectively [41–43]. IoT devices (e.g., sensors) are connected to provide end-to-end cold chain vaccine distribution. The vaccine must be stored at extremely low temperatures to remain viable. IoT platform is mainly designed to maintain vaccine temperature and authenticity of vaccine distribution in route. Generally, sensors are placed on cold containers, pallets, and vaccine packages to determine vaccine temperature during the distribution of vaccines from the warehouse to the healthcare provider. IoT platform also provides information to vaccine stakeholders along with the location details in real time.

Wayt Gibbs [57] proposed a double chain structured blockchain system for antifake and traceability vaccines. In this model, both public and private chains are integrated into the tracking platform design process and simulated in the Ethereum environment. The double chain structure provides complete information about stakeholders which includes vaccine supplier, National Medical Product Administration (NMPA), vaccine purchaser, and the vaccinated public details.

This paper presents the blockchain-based system for the anticounterfeit vaccine: reduce vaccine wastages, transparent tracking of all vaccines, storage, and delivery of the vaccine to health service providers, correctness in the registration, and ratings on vaccine based upon postvaccination side effects.

## 3. Proposed Blockchain-Based Vaccine Distribution Methodology

This section summarizes the architecture of the proposed model based on blockchain.

Vaccine supply chain management (VSCM) is a challenging aspect of the healthcare system due to critical resources, risk of counterfeit drugs, packaging errors, and lacking a product registry that may impact human life.

Vaccine vials contain delicate biological substances which need to be stored under the recommended temperature to ensure effectiveness and efficacy. The storage condition of vaccines is different. For example, Moderna requires a temperature of -20°C and is stored for up to 1 month in a normal refrigerator. On other hand, the Pfizer vaccine requires high colder temperature up to -70° and stored for up to 5 days in a normal refrigerator.

It is necessary to store the vaccine at the required temperature to maintain its efficacy. The faulty storage can be avoided with the help of blockchain. Blockchain is not owned by anyone, i.e., not centralized, but rather all the participants involved in the supply chain can join and share the information. The most critical points that need to be addressed are the process of storing, correctness in registration, distributing and monitoring vaccine vials, rating vaccine based on postvaccination side effects, and privacy of vaccinators.

In this paper, a blockchain-enabled vaccine supply chain is proposed to ensure correctness (approval of vaccine to avoid counterfeit), transparency and trust (public feedback reporting system of ramification after vaccination, storage, delivery of vaccination, and tracking of vaccine), immutable log (feedback data are protected against tampering), and the efficiency of vaccine distribution in the cold chain.

### 3.1. Design Consideration

According to the World Health Organization (WHO) report, more people died in Africa due to counterfeit drugs ordered from nonregistered vendors.

Currently, many countries are focused on anticounterfeit and ease traceability of vaccine distribution. In Africa, vaccine supply is depending on other international logistics support due to a lack of local vaccine production capacity. It makes vaccine supply very complicated to determine the source of the vaccine origin. In traditional methods, traceability of vaccine production and monitoring depends on the number labeling system. There are three major issues involved in the number labeling system: (1) numbers are easily counterfeited, (2) it is difficult to maintain the voluminous number system worldwide, and (3) immunization data is being modified or deleted [47].

The first two issues can be solved with the help of using a radio frequency identification (RFID) tag [48]. Generally, the vaccination records are maintained in the central server system which can be easily tampered with or deleted. This problem can be resolved with the help of distributed ledger system, i.e., a blockchain. The blockchain system is decentralized, and it is very hard to tamper with or delete records.

### 3.2. Vaccine Traceability and Distribution Conceptual Model

In China, the State Food and Drug Administration is responsible for the supervision and management of vaccine production. The Center for Disease Control and Prevention (CDCP) is responsible for managing the local vaccination program and purchasing vaccines from the manufacturers. CDCP distributes the vaccine to Vaccine Institution (VI). The vaccine transportation is contracted by private professional cold chain transport enterprise company.

In India, the Central Drugs Standard Control Organization (CDSCO) under the Directorate General of Health Ministry of Health & Family Welfare is responsible for transparency, accountability, and uniformity to ensure the safety, efficacy, and quality of the vaccine manufactured, imported, and distributed in the country. Government Medical Store Depots (GMSDs) procure vaccines from the manufacturers and distribute them to the regional, district, and subdistrict levels via cold-chain insulated transport enterprise.

Each country has its approval agencies for vaccination.  Figure 1 shows the system architecture of the proposed system. The application layer allows the user, vaccine manufacturers, regulatory agencies, healthcare workers, and transport enterprises in the proposed system to interact with the blockchain network. The smart contract layer is responsible for maintaining the contract for each event carried out in the network which includes code and deployment of anticounterfeit and traceability vaccine distribution. The network layer performs validation of data, consensus mechanism, and data transmission in the blockchain network. The data layer acts as a core layer that stores data in a blockchain network.

#### 3.2.1. Application Layer

The application layer is also called a physical layer which collects real-time data using Internet of Things (IoT) devices (temperature sensors, cameras, RFID tags, etc.). The vaccine is sensitive to environmental conditions. The cold chain vehicle is fixed with sensors to supervise the temperature and humidity of the vaccine during transferring the vaccine from one place to another place. The location information of transportation is updated periodically in the distributed network. All the real-time data are collected and a hash of the data is stored in the form of blocks in the network for verification.

#### 3.2.2. Contract Layer

The smart contract is a fixed set of rules which impose conformity between the two members without the involvement of third parties. In a proposed system of smart contracts, the design has five important modules. The responsibility of each module is described with the help of the following contracts: manufacturing (VM) contract, regulatory contract, transportation contract, purchase contract, and user contract.

*(1) Regulatory Contract*. The vaccine manufacturer must pass the audit before manufacturing the bulk vaccine. The manufacturer needs to perform self-checking to ensure the efficacy and safety of the vaccine. After self-testing, the manufacturer can apply for good manufacturing practice (GMP) certification from the National Regulatory Authority (NRA). If the vaccine samples pass the inspection, NRA provides the certificate for the production of the vaccine. The whole process of vaccine audit and approval process are recorded in the blockchain network.

The process of submitting vaccination registration and approval in the blockchain network is shown in Pseudocode 1. Line 1 is to check the condition of whether the proposal submitted for vaccine production and planning successfully passed the clinical trials or not. The contract is stored as a data structure in the form of a table. The role of a contract is mainly to add, query, and delete the data in a table. These operations are performed by the authorized person. The certificate authority verifies the authenticity of the drug administrator and provides credentials for the participants in the blockchain network.

*(2) Transport Contract*. The main aim of this smart contract is to build a vaccine distribution system transparently with the aid of IoT sensors and update the real-time information in the blockchain network. The vaccine manufacturer assigns some rules for the maximum and minimum temperature storage and distribution of the vaccine. The transportation of the vaccine distribution process is validated by Pseudocode 2.

*(3) Vaccinator/User Contract*. Initially, a user needs to get register with the blockchain network for vaccination. During the vaccination, the health service provider will verify the authenticity of the user and update the vaccination details in the blockchain network as given in Pseudocode 3. The user who has administrated the vaccine will give feedback about postvaccination symptoms or any side effects encountered after the vaccination.

### 3.3. Manufacturing Process

In the manufacturing process, the vaccine industries have to clear the audit of a regulatory body to carry out the manufacturing process. In the blockchain, each block stores different sorts of transactions, which are periodically updated by CLAA, VM, GMSD, HSP, and TE. Each transaction has a different data field such as a time stamp (transaction time), a sender (transaction initiator), recipient, amount of vaccine, and records of data. The vaccination data records are organized in the form of hash table structures which has unique keys and their values.

Figure 2 shows the traditional method of vaccine regulatory model. The detail of the model is as follows:

Step 1: before manufacturing the vaccine, the vaccine industry needs to submit the audit materials to the central licensing approval authority (CLAA)

Step 2: CLAA reviews the manufacturer's materials and submits the approval/rejection of vaccine production. It also assigns label numbers for a vaccine

Step 3: once the approval is received from the regulatory authorities, production activities are carried out

Steps 4-6: in each stage of vaccine distribution, all the entities such as vaccine labels and GMSD received information related to vaccines are shared with the regulatory authorities. GMSD requires verifying the vaccination details with regulatory agencies after getting the vaccine from the manufacturing unit

Step 7: HSP administrates the vaccine to the front-end users and also monitors the postvaccination effects of vaccinators and shares the information with GMSD

Step 8: GMSD shares the feedback with regulatory authorities

Figure 3 shows the architecture of the proposed vaccine distribution framework from the production of the vaccine to end delivery to the beneficiary. The main participants involved in the blockchain networks are (i) the user who will take immunization, (ii) the manufacturing industry that produces vaccine vials, (iii) sensor devices that monitor the location and temperature of cold chain supply during the distribution of vaccine and storage unit, (iv) health service provider, and (v) National Regulatory Authority that approves vaccine production. All the participants are verified by the certificate authorities, and the data is stored in distributed ledgers which are immutable and accessed by all participants. The proposed system ensures transparency at each level.

## 4. Security Analysis of Proposed System

All the participants in the system initiate the transaction once their identity is verified and validated by a certificate authority. All the users can communicate and store the transaction in the distributed ledger through the REST server composer.

### 4.1. Security against Anticounterfeit Vaccine

At present, all the information related to vaccines is stored in a centralized system in which there is a possibility of producing fake vaccines and circulating them on market.

#### 4.1.1. Proof Sketch

Pseudocode 1 in the section shows the vaccine registration and approval process of the proposed system. The proposed system maintains all the records in a decentralized system. All the information related to vaccines such as vaccine approved by drug administration, vaccine distribution, cold chain supply, vaccine distributed to a health service provider, vaccinator details, and feedback reports submitted by vaccinators is stored in the blockchain network and is immutable as well as transparent.

### 4.2. Security against Tampering of Vaccine Vials

In the current context, the vaccine management system is managed by different entities in the supply chain. The data can be easily tampered with, fudged, or deleted by any entity.

#### 4.2.1. Proof Sketch

In this proposed system, the data related to the vaccine is hoarded in blockchain with the help of consensus algorithms. Data tampering is impossible due to the huge computational power required for tampering. The security and privacy of the vaccine data can be ensured with the help of a blockchain network. Pseudocodes 2 and 3 in the section describe the how proposed system against tampering with vaccine vials during transportation and the feedback process.

## 5. Conclusions

In this paper, the blockchain-enabled vaccine supply chain mechanism is elaborated which ensures transparency of vaccine circulation, storage, transportation, delivery of vaccination, anticounterfeit vaccine, and feedback reporting after postvaccination. Blockchain network provides data immutability and verifies the transaction at each level from vaccine production to immunization campaign. The IoT devices are used to track and monitor the temperature of cold chain storage and transportation. The uniqueness of the proposed system is to provide distributed system to verify the reliability and efficacy of the vaccine from production to end beneficiaries' feedback about the vaccine. Our proposed system gives a clear view to the users as well as to the healthcare provider about the vaccination and ensures the anticounterfeit vaccine. The proposed framework will be considered for future cold chain distribution, vaccines based on the product, perseverance, and environmental constraints to minimize the distribution of counterfeit vaccine and maintain distributed vaccine records improves supply chain security and handling process. It also ensures the (i) efficacy and transparency of vaccine distribution, (ii) record related to vaccine storage and delivery, (iii) vaccinator registration details and immunization, and (iv) a transparent reporting system about the side effects. In future work, the machine learning-based recommendation engine will be integrated with the proposed system to monitor the distribution of vaccines and demand forecasting.

## Figures and Tables

**Figure 1:** System architecture of the proposed system.

**Figure 2:** Traditional vaccine regulatory model.

**Figure 3:** Architecture of proposed vaccine distribution framework.

**Pseudocode 1:** Vaccine registration and approval process.

**Pseudocode 2:** Transportation of vaccine.

**Pseudocode 3:** Feedback process.

## Data Availability

Data used in this study are available upon request.
